This article has been retracted.

# Anemia and Contributing Factors in Severely Malnourished Infants and Children Aged between 0 and 59 Months Admitted to the Treatment Centers of the Amhara Region, Ethiopia: A Multicenter Chart Review Study

**DOI:** 10.1155/2021/6636043

**Published:** 2021-03-27

**Authors:** Wubet Worku Takele, Adhanom Gebreegziabher Baraki, Haileab Fekadu Wolde, Hanna Demelash Desyibelew, Behailu Tariku Derseh, Abel Fekadu Dadi, Eskedar Getie Mekonnen, Temesgen Yihunie Akalu

**Affiliations:** ^1^Department of Community Health Nursing, School of Nursing, College of Medicine and Health Sciences, University of Gondar, Gondar, Ethiopia; ^2^Department of Epidemiology and Biostatistics, Institute of Public Health, College of Medicine and Health Sciences, University of Gondar, Gondar, Ethiopia; ^3^Department of Human Nutrition, College of Health Sciences, Bahir Dar University, Bahir Dar, Ethiopia; ^4^Department of Public Health, College of Medicine and Health Sciences, Debre Berhan University, Debre Berhan, Ethiopia; ^5^Department of Epidemiology and Biostatistics, Flinders University, Health Sciences Building, Sturt Road, Bedford Park, Adelaide, SA 5001, Australia; ^6^Departent of Reproductive and Child Health, Institute of Public Health, College of Medicine and Health Sciences, University of Gondar, Gondar, Ethiopia

## Abstract

**Background:**

Anemia among severely malnourished children is a double burden that could make the treatment outcome of severe acute malnutrition (SAM) more unfavorable. The burden and the factors are, however, uncovered among children in the Amhara region. Therefore, the study was aimed at determining the prevalence of anemia and identifying contributing factors in severely malnourished children aged between 0 and 59 months admitted to the treatment centers of the Amhara region referral hospitals.

**Methods:**

A facility-based cross-sectional study was conducted that included 1,301 infants and children, who developed SAM and were admitted to the three referral hospitals of the Amhara region. Data were extracted using a data extraction checklist. The binary logistic regression analysis was employed to show an association between the dependent and independent variables. Multicollinearity was assessed using the variance inflation factor (VIF) and no problem was detected (overall VIF = 1.67). The presence of association was declared based on the *p*-value (≤0.05), and the adjusted odds ratio with its respective 95% confidence interval was used to report the direction, as well as the strength of association.

**Results:**

About 41.43% (95% CI: 38.78%–44.13%) of severely malnourished infants and children have developed anemia, of which around half (47%) of them were under six months old. Rural residence (AOR = 1.56; 95% CI: 1.14–2.12) and HIV infection (AOR = 2.00; 95% CI: 1.04–3.86) were significantly associated with higher odds of anemia. Furthermore, being exclusively breastfed (AOR = 0.57; 95% CI 0.39–0.83) remarkably reduced the likelihood of anemia.

**Conclusions:**

This data confirms that anemia among severely malnourished infants and children is a public health problem in the Amhara region. Infants younger than six months were at a higher risk of anemia. Being a rural resident and contracting HIV infection have elevated the occurrence of anemia, whereas being exclusively breastfed decreased the risk. Therefore, the study gives an insight to policymakers and planners to strengthen the existing exclusive breastfeeding practice. Strategies being practiced to prevent HIV transmission and early detection, as well as treatment, should also be strengthened. Furthermore, mothers/caretakers of infants and children residing in the rural areas deserve special attention through delivering nutrition education.

## 1. Introduction

Anemia contributes to a wide range of health problems like heart failure, poor cognitive performance, and macro- and micronutrient deficiencies [1, 2]. The burden is the third top-ranked childhood cause of death, which accounted for 8.1% of the total mortalities [3]. Anemia is a hematological disorder that occurs in individuals of all ages though it is most prevalent and severe among reproductive-age women, children younger than five years, sick children, and children suffering from other nutritional deficiency disorders [4]. A sufficient hemoglobin concentration in the human blood is an important indicator of the availability of enough trace minerals, especially iron, as it is a precursor for the synthesis of hemoglobin, which is an important messenger that transports crucial nutrients and oxygen to different parts of the body [5]. A hemoglobin concentration below 11 g/dl is defined as anemia [6]. Anemia is associated with micronutrient deficiencies such as vitamin B-12 and B-9, as well as different infectious diseases that primarily attack the red blood cells [7, 8]. Likewise, iron deficiency shares 50% of all causes of anemia, and it is basically linked with poor dietary intake [9].

SAM and anemia have aninterply association [10, 11]. In other words, childhood anemia might occur as a result of macronutrient deficiency (particularly protein), or it precipitates the occurrence of undernutrition owing to the poor synthesis of macronutrients notably protein [9, 10, 12]. Worldwide, about 18.7 million children are severely malnourished and have prominent micronutrient deficiency, of which 18.5 million are from lower- and middle-income countries [13]. SAM is characterized by the presence of bilateral pitting edema and severe wasting (weight-for-height/length 70%/<−3 standard deviation) and mid upper arm circumference (MUAC) of below 11.5 cm (children older than 6 months) [14]. The concurrent occurrence of anemia and SAM makes the management process more complicated and escalates the likelihood of death. Anemia is indeed the commonest comorbid medical problem seen in children suffering from SAM and commonly referred to as “complicated SAM,” which prolongs the recovery time and increases the likelihood of mortality compared with anemic children without SAM and nonanemic children with SAM [15–18]. Surprisingly, the prevalence of anemia among this population ranges from 81.1% to 95% [1, 15, 19]; and in Ethiopia, it is estimated to be between 16.4% and 61.3% [18, 20–22].

In cognizant of the observed nutritional problem among infants and children, Ethiopia is working on improving childhood nutrition through designing various strategies like 1000 days (conception time through to two years of age), Essential Nutrition Action (ENA), Seqota Declaration, and National Nutrition Program (NNP). However, the available studies are not sufficient and thus the role of repeated scientific investigations is significant to show the burden of the problem and contributing factors.

Therefore, a summarized figure that could reflect the burden of anemia and contributing factors among severely malnourished infants and children is imperative to pass a sound decision. In doing so, it would be possible to urge the responsible bodies to recognize the issue and exert appropriate actions to strengthen the strategies that are in place. Similarly, programmers may use this finding as an implementation evaluation. Moreover, the results of this study would stimulate clinicians to stringently follow infants and children suffering from SAM and apply appropriate interventions as early as possible.

## 2. Methods

### 2.1. Study Design, Period, and Setting

An institution-based cross-sectional study was conducted among infants and children who were hospitalized between October 2012 and September 2016 at inpatient SAM treatment centers of the Amhara region referral hospitals. Data were gathered from the three hospitals of the region: the University of Gondar, Debre Berhan, and Felege Hiwot referral hospitals. Clinicians working in these hospitals are recommended to follow the national treatment protocol while admitting and treating infants and children. Furthermore, these hospitals have separate inpatient treatment centers whereby severely malnourished children are admitted and receive appropriate nutritional and medical care.

### 2.2. Study Population and Sample

The study considered all severely malnourished infants and children who were admitted to the SAM inpatient treatment centers of the three aforementioned hospitals. Only children whose anemic status was diagnosed using a hemoglobin test at admission, or before starting the transition phase management, were recruited. This is because children who are at the transition phase obviously start to receive therapies like ready-to-use therapeutic feeding (RUTF), which has trace minerals and could affect the estimation. About 401, 373, and 527 participants were from Felege Hiwot, Debre Berhan, and University of Gondar referral hospitals, respectively, making a total sample size of 1,301.

### 2.3. Variables of the Study

The outcome variable was anemia and it was ascertained biochemically using hemoglobin status. Sociodemographic factors, such as the health facility's name, children's sex, children's age, and residence were included. Breastfeeding status, vaccination status, presence of diarrhea, presence of pneumonia, type of SAM, HIV status, antibiotic intake, folic acid supplementation, and vitamin A supplementation were the independent variables.

### 2.4. Anemia and Anthropometry Measurements

Infants and children whose hemoglobin concentration was below 11 g/dl were labeled as anemic [6]. Although the abovementioned criterion is for infants and children younger than six months, the same cut-off point was used for children older than six months, as there is no other standard for this group of population and it is commonly applicable in the clinical set-up [23].

Infant's and children's nutritional status was measured using the national guideline for management of SAM. Accordingly, SAM was diagnosed as either the presence of severe wasting (weight-for-height/length 70%/<−3 SD) or bilateral pitting edema of both feet or MUAC of below 11.5 cm (for only children older than six months) [14, 24].

### 2.5. Breastfeeding and Immunization Status

Breastfeeding status was taken from the chart and children who were breastfed for the first six months without adding other foods other than the prescribed medicines were considered as exclusively breastfed [25]. Immunization status was explained as “unimmunized,” “fully immunized,” “unknown,” and “incomplete,” according to the World Health Organization (WHO) [26]. Children who did not receive any vaccine during their immunization period were considered “unimmunized,” according to the evidence recorded in the medical recordings. Infants and children who had missed receiving at least one of the recommended vaccines were categorized as “incompletely immunized,” whereas “fully vaccinated” was defined as infants and children who have completed and received the vaccine according to their age. Unknown vaccination status was declared when there was no vaccination history recorded in the medical record. However, for infants younger than 12 months, their immunization status was considered as “fully immunized” provided that they received age-appropriate vaccines, and it was considered “incomplete” if they missed one of the immunization schedules.

### 2.6. Clinical Forms of Malnutrition

The types of SAM were described using the clinical presentations[27]. Accordingly, infants and children who had no edema but had fat wastage and other supplementary clinical presentations diagnosed with marasmus. Infants and children who had edema, muscle wastage, and other clinical manifestations were diagnosed with kwashiorkor. Lastly, infants and children who had mixed forms of clinical presentations of the abovementioned malnutrition forms were diagnosed as having both marasmus and kwashiorkor.

### 2.7. HIV and Tuberculosis Infection

The HIV infection status was considered using the confirmatory tests as per the national test algorism of the country. Infants and children aged under eighteen months had their HIV status examined using polymerization chain reaction (PCR) and those whose results were positive were assigned the status positive for HIV infection, whereas children older than eighteen months had their HIV status examined using any confirmatory antibody test and those whose results were positive were assigned the status positive for HIV infection [28]. Similarly, only confirmed tuberculosis (TB) infection was considered.

### 2.8. Data Collection Procedure, Quality Assurance, and Extraction Procedure

The data were collected using a data extraction sheet comprised of all independent and dependent variables. Prior to the commencement of the data collection, training of two days was given for two data collectors and one supervisor in each hospital aiming at briefing about the objectives of the study and what kind of data should be extracted. A pretest was performed in order to understand the variables that are available in the medical registering chart. Data reported the hemoglobin status analyzed through HemaCue-HB 201, and hematological analyzer machine was considered. The completeness of the data was checked on a daily basis. Finally, the data sets from the three hospitals were merged.

### 2.9. Data Processing and Analysis

The collected data were entered into Epi-data version 4.4.3.1 and exported to STATA version 14, and coding, cleaning, and analyses were done accordingly. All continuous independent variables were categorized. The outcome variable was dichotomized and coded as “0” and “1,” representing not anemic and anemic, respectively. For continuous variables, such as age, the histogram was used to determine which measure of central tendency is appropriate. Descriptive statistics such as frequency, percentages, and measures of central tendency with their appropriate corresponding measure of dispersion were used. Tables and texts were used to present the findings.

Furthermore, the binary logistic regression analysis was applied to identify factors associated with anemia. Variables with a *p* value of less than 0.2 in the bivariable analysis were transferred to multivariable analysis to control the possible effects of confounder/s and identify the significant variables. Hosmer and Lemeshow goodness-of-fit test was used to examine the model adequacy, and it was insignificant (*p*  value= 0.79).

The interaction of independent variables was checked by a multicollinearity test using the variance inflation factor (VIF), and no problem was detected (overall VIF = 1.67). Finally, the presence of an association between the independent and dependent variables and its direction and strength were established by the AOR with its corresponding 95% CI for variables with *p*-value <0.05. The difference in outcome among hospitals was checked by intraclass correlation (ICC), and no significant difference was observed. As a result, the model without considering variability was used.

### 2.10. Ethical Consideration

Ethical clearance was obtained from the ethical review committee of the three referral hospitals, and a permission letter was also obtained from the respective hospitals. As the study was conducted through a review of records, no consent was asked from the mothers, or caregivers of the study subjects. The confidentiality and privacy of the patient record was ensured by avoiding names and identification number from extraction form and using codes instead.

## 3. Results

### 3.1. Sociodemographic Characteristics of Children with SAM

The medical records of 1,301 children with SAM were reviewed. The median age of children was 16 months (interquartile range (±IQR) of 9 to 24 months). Of all respondents, 527 (40.51%) were from the University of Gondar referral hospital. More than half (54.57%) of children were females and nearly two-thirds (64.43%) of them were from rural residence. A small proportion (6%), two-fifths (40%), and just over one-third (33.59%) of them were fully vaccinated, had developed diarrhea, and contracted pneumonia, respectively. One hundred seven (8.22%) and 54 (4.15%) children with SAM had TB and HIV, respectively. Moreover, just more than four of every ten (42.86%) children took antibiotics, while 65.82% were supplemented with folic acid (Table 1).

### 3.2. Prevalence of Anemia

The prevalence of anemia among under-five-year-old infants and children suffering from SAM was 41.43%, 95% CI: (38.78%, 44.13%). The magnitude varied throughout the age categories and a third of severely malnourished infants and children younger than six months were anemic: 36.15%, 95% CI: (27.92%, 45.04%). Furthermore, nearly equal proportion of them aged 6–23 months and ≥23 months had experienced anemia: 41.73% (95% CI: 38.42, 45.10) and 42.81% (95% CI: 37.19, 48.56), respectively.

### 3.3. Factors Associated with Anemia

In the bivariable logistic regression analysis, age, residence, exclusive breastfeeding, type of SAM, pneumonia, tuberculosis infection, HIV status, taking antibiotics, and supplemented vitamin A were entered into a multivariable logistic regression model. After the adjustment, residence, exclusive breastfeeding, and HIV status remained significantly associated with anemia.

The odds of anemia among rural dwellers was 56% higher than urban residents (AOR = 1.56; 95% CI: (1.14, 2.12)). Similarly, infants and children who had contracted HIV infection were two times higher to develop anemia compared with their counterparts (AOR = 2.00; 95% CI: (1.04–3.86)). The odds of anemia among exclusively breastfed children was decreased by 43%, compared with their nonexclusively breastfed counterparts (AOR = 0.57; 95%CI: (0.39, 0.83)) (Table 2).

## 4. Discussion

Malnutrition is a lingering and important public health problem, affecting the lives of multiple children and women in developing countries like Ethiopia. Anemia is an auxiliary nutritional problem that could interfere with recovery from illness. Carrying out studies among this disadvantaged population is imperative to understand the problem and take corrective measures accordingly. Hence, the aim of this study was to assess the prevalence of anemia and factors among under-five-year-old children with SAM in the Amhara region.

The prevalence of anemia among children with SAM aged between 0 and 59 months was 41.43% (38.78%–44.13%), which is a public health pressing problem requiring urgent attention of clinicians and policymakers. The finding is lower than that of a study from Vavuniya, Sri Lanka (55.5%) [29]. Sir Lanka's study was done in a single rural district (Vavuniya), in which more than 70% of children with SAM were from a socially deprived society. However ththe current study is mainly conducted in cities presumably wealthier although there was some possibility of incorporating referral cases from rural areas. Similarly, the finding of the study is lower than a study from Turbo, Columbia (51.1%) [30]. This could be due to the inclusion of children under six months old in the current study, who are at a lower risk of being anemic compared with children older than six months [31, 32].

This finding is also lower than that of a study from Guinea-Bissau (80.2%) [1]. Guinea-Bissau's study was conducted in a rural area in which most children would have a greater possibility of working in agricultural areas which create a potential risk of acquiring soil-transmitted hookworm infections that could increase the risk of anemia [33].

As far as factors contributing to anemia is concerned, rural residence, being exclusively breastfed, and having HIV infection contributed to the development of anemia. The study highlighted that rural residence was associated with higher odds of anemia, depicting that those rural children are disadvantageous over their peers residing in an urban area in experiencing extra nutritional complications, including (but are not limited to) macro and micronutrient deficiencies that could lead to death [34]. Studies have shown that the sequelae of anemia are diversified like deficiencies of other important micronutrients and extra nutrition problems [35]. Consequently, these children could encounter poor neurodevelopment and are incapable of carrying out tasks demanding cognitive performance [2, 36]. This finding is supported by a multicenter study from Burkina Faso, Ghana, and Mali [37]. Furthermore, a study from Uganda showed that rural residence introduced a higher risk of anemia due to poor access to health services, including health education [38], which would help residents maintain their self and environmental hygiene. Additionally, the poor availability and accessibility of nutrient-rich food items in the area related to food insecurity and other attributes [39].

The current data suggest that exclusive breastfeeding decreases the odds of anemia. Alternatively, previous studies revealed that the duration of exclusive breastfeeding is one of the risk factors for the ongoing development of anemia [40]; the longer the duration of breastfeeding, the higher the risk of experiencing anemia. Likewise, existing literature speculated that exclusive breastfeeding contributes to developing anemia; it is known that as the child grows, the nutrient requirements become higher, and the infant iron storage acquired from the mother through the placenta become depleted, which might not be compensated by the breast milk only as it contains a small amount of iron [41, 42]. To that end, studies suggest that supplementing iron at this stage could limit the development of childhood anemia [43, 44]. Taking all the arguments in the current and the previous studies into consideration, further investigations that involve high-level studies are highly recommended.

Furthermore, HIV infection has doubled the odds of developing anemia. There are a wide range of mechanisms to how HIV infection could lead to anemia: it results in excessive RBC destruction and ineffective RBC production as a result of invading the hematopoiesis sites such as bone marrow [45–47]. The other mechanism is that the infection reduces the erythropoietin performance [48, 49]. Likewise, some antiretroviral therapy (ART) drugs like zidovudine (AZT) usually cause anemia by interfering with the production of RBCs [50, 51]. The cell proliferation of organs in this segment of the population is less competitive compared with healthy counterparts. Furthermore, vitamin B12, an indispensable vitamin that supports the role of iron in the synthesis of hemoglobin, is deficient among HIV-infected individuals [52]. This vitamin deficiency is commonly seen in malnourished individuals secondary to gastric malfunction and the problem is a vicious cycle. Therefore, it is possible to draw an inference that HIV infection worsens childhood anemia among children with SAM because of the dual effects of poor RBC production and the deleterious effect of AZT. The study implies that apart from weakening the immunity and opening a great opportunity for other opportunistic infections, HIV infection jeopardizes the body's capability of generating RBCs and the production of hemoglobin. In addition, HIV infection shortens the lives of individuals, and it is notable that this infection would significantly reduce the survival of children with SAM. Thus, to limit the occurrence of opportunistic infection and facilitate the RBC production, which are both significant to prevent anemia, early treatment and prevention of HIV infection is recommended as usual.

Considering that multicentered sites of the region could reflect the strength of the study and thus could fortify the generalizability of the findings to the region. Similarly, as the data were gathered from different sites, the study considered a clustering effect. However, this study was based on secondary data; therefore, the study suffered from incomplete data, and as a result, some charts of the children were not considered.

## 5. Conclusions

The study suggests that just greater than a third of severely malnourished children aged between 0 and 59 months admitted to the treatment centers of the Amhara region referral hospitals have developed anemia, echoing a public health problem. Being a rural resident and having an HIV infection have elevated the occurrence of anemia, whereas exclusive breastfeeding reduced the likelihood. Therefore, it is valuable for policymakers and planners to strengthen the preventive strategies of HIV infection and give a special focus to rural residents. In addition, clinicians working in maternal and child health departments are recommended to strengthen the treatment of HIV infection before causing further damages. Although the current study has come up with evidence revealing the protective effect of exclusive breastfeeding on anemia, it contradicts the existing literature and it is quite impossible to draw a conclusion basing this study. Therefore, future scholars are recommended to conduct a study that helps solve the observed contradiction.

## Figures and Tables

**Table 1:** Sociodemographic characteristics of children with SAM in the Amhara region, northwest Ethiopia, 2016.

Variables	Frequency	Percentage
Location of health facility		
Felege Hiwot Referral Hospital	401	30.82
Debre Berhan Referral Hospital	373	28.67
Gondar Referral Hospital	527	40.51
Child's sex		
Male	591	45.43
Female	710	54.57
Child's age		
Under 6 months	130	9.99
6–23 months	865	66.49
2 years and above	306	23.52
Residence		
Rural	837	64.43
Urban	462	35.57
Exclusive breastfeeding		
No	241	18.52
Yes	1,060	81.48
Immunization status		
Unimmunized	90	6.92
Incompletely immunized	495	38.05
Fully immunized	81	6.23
Unknown	635	48.80
Diarrhea		
No	794	61.03
Yes	507	38.97
Pneumonia		
No	864	66.41
Yes	437	33.59
Type of SAM		
Marasmus	888	68.26
Kwashiorkor	273	20.98
Marasmus and kwashiorkor	140	10.76
Tuberculosis		
Yes	107	8.22
No	1,194	91.78
HIV status		
Positive	54	4.15
Negative	885	68.02
Unknown	362	27.82
Antibiotics		
Given	393	42.86
Not given	524	57.14
Folic acid		
Given	859	65.82
Not given	446	34.18
Vitamin A		
Given	763	83.30
Not given	153	16.70

**Table 2:** Factors associated with anemia among children with SAM aged 0–59 months in the Amhara regional state, northwest Ethiopia, 2016.

Variables	Anemia		COR (95% CI)	AOR (95% CI)	*p* value
	Yes	No			
Age					
<24 months	333	504	1	1	
≥24 months	205	257	1.21 (0.96, 1.52)	1.08 (0.81,1.45)	0.34
Residence					
Rural	300	372	1.51 (1.12, 2.04)	1.56 (1.14, 2.12)	0.031
Urban	89	167	1.	1	
Exclusively breastfed					
No	121	120	1	1	
Yes	418	642	0.65 (0.49, 0.86)	0.57 (0.39, 0.83)	0.02
Type of SAM					
Marasmus	334	554	1	1	
Kwashiorkor	140	133	1.75 (1.33, 2.29)	1.12 (0.76, 1.63)	0.43
Marasmus and kwashiorkor	65	75	1.44 (1.01, 2.06)	1.24 (0.81, 1.89)	0.31
Pneumonia					
Absent	371	493	1	1	
Present	168	269	0.83 (0.66, 1.05)	0.87 (0.64, 1.22)	0.11
Tuberculosis					
No	488	706	1	1	
Yes	51	56	1.32 (0.89, 1.96)	1.38 (0.87, 2.19)	0.21
HIV					
Negative	355	530	1	1	
Positive	31	23	2.01 (1.15, 3.51)	2.00 (1.04, 3.86)	0.01
Unknown	153	209	1.09 (0.85, 1.40)	1.03 (0.72, 1.46)	0.22
Antibiotics					
Given	181	212	1.31 (1.01, 1.72)	1.25 (0.93, 1.66)	0.35
Not given	206	318	1	1	
Vitamin A					
Not given	133	151	1	1	
Given	254	379	0.76 (0.57, 1.01)	0.86 (0.63, 1.19)	0.37

## Data Availability

All the relevant data used to present the study are available; however, the corresponding author will supply the data upon request.

## Abbreviation

AIDS: Acquired Immunodeficiency Syndrome
AOR: Adjusted odds ratio
COR: Crude Odds Ratio
CI: Confidence Interval
HIV: Human Immunodeficiency Virus
IQR: Interquartile Range
MUAC: Midupper Arm Circumference
SAM: Severe Acute Malnutrition
SD: Standard Deviation
TB: Tuberculosis
WHO: World Health Organization
WHZ: Weight-for-Height *Z* Score.

## References

[1] Thorne C. J., Roberts L. M., Edwards D. R., Haque M. S., Cumbassa A., Last A. R. (2013). Anaemia and malnutrition in children aged 0-59 months on the Bijagós Archipelago, Guinea-Bissau, West Africa: a cross-sectional, population-based study. *Paediatrics and International Child Health*.

[2] Halterman J. S., Kaczorowski J. M., Aligne C. A., Auinger P., Szilagyi P. G. (2001). Iron deficiency and cognitive achievement among school-aged children and adolescents in the United States. *Pediatrics*.

[3] Related H PE. Federal Ministry of Health Health and Health Related Indicators. 2005 E.C (2012/2013). 2014

[4] Stoltzfus R. J., Chwaya H. M., Tielsch J. M., Schulze K. J., Albonico M., Savioli L. (1997). Epidemiology of iron deficiency anemia in Zanzibari schoolchildren: the importance of hookworms. *The American Journal of Clinical Nutrition*.

[5] Allen L. H., Rosado J. L., Casterline J. E. (2000). Lack of hemoglobin response to iron supplementation in anemic Mexican preschoolers with multiple micronutrient deficiencies. *The American Journal of Clinical Nutrition*.

[6] World Health Organization (2011). *Haemoglobin Concentrations for the Diagnosis of Anaemia and Assessment of Severity. Vitamin and Mineral Nutrition Information System*.

[7] Duque X., Flores S., Flores-Huerta S., Mendez-Ramirez I., Munoz S. (2007). Prevalence of anemia and deficiency of iron folic acid and zinc in children under 2 years of age and beneficiaries of the Mexican Social Security Institute. *BMC Public Health*.

[8] Schneider J. M., Fujii M. L., Lamp C. L., Lönnerdal B., Dewey K. G., Zidenberg-Cherr S. (2005). Anemia, iron deficiency, and iron deficiency anemia in 12-36-mo-old children from low-income families. *The American Journal of Clinical Nutrition*.

[9] World Health Organization (1968). *Nutritional Anaemias: Report of a WHO Scientific Group (Meeting Held in Geneva from 13 to 17 March 1967)*.

[10] Guerrant R. L., Oriá R. B., Moore S. R., Oriá M. O., Lima A. A. (2008). Malnutrition as an enteric infectious disease with long-term effects on child development. *Nutrition Reviews*.

[11] Ehrhardt S., Burchard G. D., Mantel C. (2006). Malaria, anemia, and malnutrition in african children-defining intervention priorities. *The Journal of Infectious Diseases*.

[12] Kahigwa E., Schellenberg D., Sanz S. (2002). Risk factors for presentation to hospital with severe anaemia in Tanzanian children: a case-control study. *Tropical Medicine and International Health*.

[13] Black R. E., Victora C. G., Walker S. P. (2013). Maternal and child undernutrition and overweight in low-income and middle-income countries. *The Lancet*.

[14] World Health Organization (2007). *UNICEF: Community-Based Management of Severe Acute Malnutrition: A Joint Statement by the World Health Organization, the World Food Programme, the United Nations System Standing Committee Onnutrition and the United Nations Children’s Fund*.

[15] Dwivedi D., Singh V., Singh J., Sharma S. (2017). Study of anaemia in children with severe acute malnutrition. *Journal of Nepal Paediatric Society*.

[16] Girum T., Kote M., Tariku B., Bekele H. (2017). Survival status and predictors of mortality among severely acute malnourished children <5 years of age admitted to stabilization centers in Gedeo Zone: a retrospective cohort study. *Therapeutics and Clinical Risk Management*.

[17] Jarso H., Workicho A., Alemseged F. (2015). Survival status and predictors of mortality in severely malnourished children admitted to Jimma University Specialized Hospital from 2010 to 2012, Jimma, Ethiopia: a retrospective longitudinal study. *BMC Pediatrics*.

[18] Wagnew F., Dejenu G., Eshetie S., Alebel A., Worku W., Abajobir A. A. (2019). Treatment cure rate and its predictors among children with severe acute malnutrition in Northwest Ethiopia: a retrospective record review. *PLoS One*.

[19] Thakur N., Chandra J., Pemde H., Singh V. (2014). Anemia in severe acute malnutrition. *Nutrition*.

[20] Gelaw T. T., Wondemagegn A. M. (2013). Response to conventional nutritional treatment of severely malnourished hospitalized children in the context of HIV infection at Yekatit 12 hospital, Addis Ababa, Ethiopia. *Science Journal of Clinical Medicine*.

[21] Derseh B., Mruts K., Demie T., Gebremariam T. (2018). Co-morbidity, treatment outcomes and factors affecting the recovery rate of under-five children with severe acute malnutrition admitted in selected hospitals from Ethiopia: retrospective follow up study. *Nutrition Journal*.

[22] Ahmed M. (2014). *Managment Outcome of Severe Acute Malnutrition from 6 Months to 5 Years of Age Children Admitted to Yekatit 12 Hospital*.

[23] Wintrobe M., Lee G. R., Bogs T. R. (1981). *Clinical Hematoloty*.

[24] World Health Organization (2013). *Guideline: Updates on the Management of Severe Acute Malnutrition in Infants and Children*.

[25] World Health Organisation (1991). *Indicators for Assessing Breastfeeding Practices: Report of an Informal Meeting*.

[26] World Health Organization (2017). *Immunization, Vaccines, and Biologicals: Implementation Research in Immunization*.

[27] den Broeck Van J., Meulemans W., Eeckels R. (1994). Nutritional assessment: the problem of clinical-anthropometrical mismatch. *European Journal of Clinical Nutrition*.

[28] Read J. S. (2007). Diagnosis of HIV-1 infection in children younger than 18 months in the United States. *Pediatrics*.

[29] Keerthiwansa J., Gajealan S., Sivaraja S., Subashini K. (2014). Malnutrition and anaemia among hospitalised children in Vavuniya. *Ceylon Medical Journal*.

[30] Bernal C., Velásquez C., Alcaraz G., Botero J. (2008). Treatment of severe malnutrition in children: experience in implementing the World Health Organization guidelines in Turbo, Colombia. *Journal of Pediatric Gastroenterology & Nutrition*.

[31] Monteiro C. A., Szarfarc S. C., Mondini L. (2000). Tendência secular da anemia na infância na cidade de São Paulo (1984–1996). *Revista de Saúde Pública*.

[32] Assis A. M. O., Gaudenzi E. N., Gomes G., Ribeiro R. D. C., Szarfarc S. C., Souza S. B. D. (2004). Hemoglobin concentration, breastfeeding and complementary feeding in the first year of life. *Revista de Saúde Pública*.

[33] Svedberg P. (1990). Undernutrition in Sub‐Saharan Africa: is there a gender bias?. *Journal of Development Studies*.

[34] Wagnew F., Dessie G., Takele W. W. (2019). A meta-analysis of inpatient treatment outcomes of severe acute malnutrition and predictors of mortality among under-five children in Ethiopia. *BMC Public Health*.

[35] Azab S. F. A., Abdelsalam S. M., Saleh S. H. A. (2014). Iron deficiency anemia as a risk factor for cerebrovascular events in early childhood: a case-control study. *Annals of Hematology*.

[36] Baker R. D., Greer F. R. (2010). Diagnosis and prevention of iron deficiency and iron-deficiency anemia in infants and young children (0–3 years of age). *Pediatrics*.

[37] Magalhães R. J., Clements A. C. (2011). Mapping the risk of anaemia in preschool-age children: the contribution of malnutrition, malaria, and helminth infections in West Africa. *PLoS Medicine*.

[38] Kuziga F., Adoke Y., Wanyenze R. K. (2017). Prevalence and factors associated with anaemia among children aged 6 to 59 months in Namutumba district, Uganda: a cross-sectional study. *BMC Pediatrics*.

[39] Greffeuille V., Sophonneary P., Laillou A. (2016). Persistent inequalities in child undernutrition in Cambodia from 2000 until today. *Nutrients*.

[40] Marques R. F. S. V., Taddei J. A. A. C., Lopez F. A., Braga J. A. P. (2014). Breastfeeding exclusively and iron deficiency anemia during the first 6 months of age. *Revista da Associação Médica Brasileira*.

[41] Burke R. M., Rebolledo P. A., Aceituno A. M. (2018). Effect of infant feeding practices on iron status in a cohort study of Bolivian infants. *BMC Pediatrics*.

[42] Maria de Lourdes P., Lira P. I., Coutinho S. B., Eickmann S. H., Lima M. C. (2010). Influence of breastfeeding type and maternal anemia on hemoglobin concentration in 6-month-old infants. *Jornal de Pediatria*.

[43] Dijkhuizen M. A., Wieringa F. T., West C. E., Martuti S., Muhilal (2001). Effects of iron and zinc supplementation in Indonesian infants on micronutrient status and growth. *The Journal of Nutrition*.

[44] Shakur Y. A., Choudhury N., Ziauddin Hyder S., Zlotkin S. H. (2010). Unexpectedly high early prevalence of anaemia in 6-month-old breast-fed infants in rural Bangladesh. *Public Health Nutrition*.

[45] Volberding P. A., Levine A. M., Dieterich D. (2004). Anemia in HIV infection: clinical impact and evidence-based management strategies. *Clinical Infectious Diseases*.

[46] Cleveland R., Liu Y. (1996). CD4 expression by erythroid precursor cells in human bone marrow. *Blood*.

[47] Ciaffoni S., Luzzati R., Roata C., Turrini A., Antonello O., Aprili G. (1992). Presence and significance of cold agglutinins in patients with HIV infection. *Haematologica*.

[48] Spivak J. L., Barnes D. C., Fuchs E., Quinn T. C. (1989). Serum immunoreactive erythropoietin in HIV-infected patients. *The Journal of the American Medical Association*.

[49] Pfeiffer C. J. (1970). Gastrointestinal response to malnutrition and starvation. *Postgraduate Medicine*.

[50] Sperling R. (1998). Effect of ART drug ZDV (zidovudine). *Infectious Diseases in Obstetrics and Gynecology*.

[51] Dash K. R., Meher L. K., Hui P. K., Behera S. K., Nayak S. N. (2015). High incidence of zidovudine induced anaemia in HIV infected patients in Southern Odisha. *Indian Journal of Hematology and Blood Transfusion*.

[52] Remacha A. F., Rierasp A., Cadafalch J., Gimferrer E. (1991). Vitamin B‐12 abnormalities in HIV‐infected patients. *European Journal of Haematology*.

